# Genetic analysis of a patient with coexisting acromegaly, thyroid papillary carcinoma and subcutaneous fibroma

**DOI:** 10.3892/ol.2014.2824

**Published:** 2014-12-23

**Authors:** JINGFANG LIU, XULEI TANG, JIANGUO CHENG, LITING WANG, XIAOMEI YANG, YAN WANG

**Affiliations:** Department of Endocrinology, The First Hospital of Lanzhou University, Lanzhou, Gansu 730000, P.R. China

**Keywords:** acromegaly, pituitary adenomas, multiple endocrinologic neoplasia syndrome 1, *MEN1*, gsα

## Abstract

The aim of the present study was to analyze the *MEN1* and gsα gene mutations in a Chinese patient with growth hormone-producing pituitary tumors causing acromegaly, papillary thyroid carcinoma and subcutaneous fibroma. Genomic DNA was isolated from the patient and 10 healthy controls, and prepared for polymerase chain reaction (PCR) analysis. Numerous pairs of primers were designed to amplify exons 1–10 of the *MEN1* gene and exons 8 and 9 of the gsα gene, and the PCR products were sequenced to detect mutations. In the study patient, a heterozygous G→A mutation was detected at nucleotide 7848 within exon 10 of the *MEN1* gene; the missense mutation caused the substitution of alanine with threonine at amino acid 541 (A541T) in the menin protein. In addition, a G→A mutation at nucleotide 7997 within exon 10 of the *MEN1* gene was identified; the mutation was synonymous, therefore, the proline at amino acid 590 of the menin protein (P590P) did not change. No other mutations were observed in exons 8 and 9 of the gsα gene, therefore, the G7848A mutation within exon 10 of the *MEN1* gene may represent the molecular pathology underlying pituitary somatotroph adenomas and papillary thyroid carcinoma. Furthermore, the pituitary adenomas, thyroid carcinoma and subcutaneous fibroma of the present patient may be considered as early manifestations of multiple endocrinologic neoplasia syndrome 1 as opposed to pure endocrine tumors, however, a long-term follow-up study is required to clarify this.

## Introduction

Pituitary adenomas are a relatively common type of intracranial neoplasm, however, the mechanisms underlying its pathogenesis have yet to be fully elucidated. Genetic alterations, such as missense mutations in the gene-encoding α-subunit of G protein (gsα) or the *MEN1* gene in multiple endocrinologic neoplasia syndrome 1 (MEN1) have been identified in pituitary adenomas (1–5).

Gsα mutations have been identified in growth hormone (GH)-secreting pituitary adenomas and non-functioning pituitary adenomas. These mutations include the replacement of arginine by cysteine, serine or histidine in codon 201 of exon 8, or the replacement of glutamine by arginine or leucine in codon 227 of exon 9 (1,6,7). Furthermore, a previous study reported that the frequency of gsα mutations in patients with GH-secreting pituitary adenomas ranged between 4.4 and 43% (2,3).

Patients with MEN1 are predisposed to developing tumors of the parathyroid, pancreas and pituitary gland. The disease is caused by inactivating mutations in *MEN1,* a putative tumor suppressor gene, which has been localized to chromosome 11q13 by genetic mapping studies (8). Loss of heterozygosity has been identified in *MEN1*-associated pituitary adenomas and in 10–18% of sporadic pituitary adenoma patients, indicating the involvement of *MEN1* (9). Furthermore, a significant proportion of sporadic pituitary tumors harboring deletions map to the critically deleted region of the *MEN1* gene (4). The present study describes the case of a female patient with a coexisting GH-producing pituitary tumor, papillary thyroid carcinoma and subcutaneous fibroma. Despite surgery, Gamma-Knife^®^ radiosurgery and octreotide acetate treatment of the GH-producing pituitary tumor, the patient’s GH levels remained elevated, with no evidence of residual pituitary tumor on a computed tomography scan. Thus, the germinal mutations in the *MEN1* and gsα genes were analyzed to investigate the molecular pathology of the tumors. Written informed consent was obtained from the patient.

## Patient and methods

### Case report

In September 2012, a 39-year-old female presented to the Department of Endocrinology, The First Hospital of Lanzhou University (Lanzhou, China) with progressive enlargement of the hands, feet and lips for 12 years. In June 2000, the patient presented with typical manifestations of acromegaly, including progressive enlargement of the hands, feet, lip and tongue, pachylosis and sleep apnea. In April 2007, the patient underwent surgery to remove a nodule in the left shoulder, which was histopathologically diagnosed as a subcutaneous fibroma. In March 2009, magnetic resonance imaging revealed a pituitary macroadenoma with a GH level of >40 ng/ml. The patient underwent a pituitary adenoma resection via the single nostril transsphenoidal approach, and subsequent pathological analysis of the tumor was consistent with a pure, densely granulated, GH-producing pituitary adenoma (somatotropinoma). In addition, in August 2009 and March 2012, the patient underwent Gamma-Knife radiosurgery for the treatment of residual tumor detected by a computed tomography scan and for persistent acromegaly with GH levels of >20 ng/ml, respectively. However, three months after Gamma-Knife treatment, the patient’s GH levels increased to 21.2 ng/ml.

Finally, in November 2011, cervical ultrasonography revealed a 1.3×1.8-cm, irregular-shaped nodule on the left posterior lobe of the thyroid and a 1.1×0.8-cm, irregular-shaped nodule on the right lobe of the thyroid. The patient therefore underwent a total thyroidectomy and ipsilateral level VI lymph node dissection. Subsequent histopathological analysis revealed a left thyroid papillary carcinoma, which was negative for RET expression, therefore, levothyroxine was administered orally at a dose of 150 μg/day following thyroid surgery.

In September 2012, a physical examination indicated a blood pressure of 110/68 mmHg, and acromegaly manifesting as prognathism, a prominent forehead, flat nose and macroglossia. Furthermore, mild anemia without jaundice and no lymphadenopathy were observed.

The results of the laboratory analyses that were conducted are summarized in Table I. Thyroid function tests indicated the following levels: Thyroid-stimulating hormone, 0.229 μIU/ml (normal range, 0.55–4.78 μIU/ml); triiodothyronine (T_3_), 1.02 ng/ml (normal range, 0.60–1.81 ng/ml); thyroxine (T_4_), 10.50 μg/dl (normal range, 4.50–10.90 μg/dl); free(F)T_3_, 3.33 pg/ml (normal range, 2.3–4.2 pg/ml); FT_4_, 1.73 ng/dl (normal range, 0.89–1.76 ng/dl); and thyroglobulin, <0.1mg/ml. Additionally, the GH level was 23.94 ng/ml (nadir GH level following glucose load of 19.57 ng/ml) and the insulin-like growth factor level was 1103 ng/ml (normal range, 570±25 ng/ml). The sex hormone, adrenocorticotropic hormone, cortisol and prolactin levels were within the normal ranges, and the bone mineral density at the calcaneus was 0.154 g/cm^2^ (normal range, >0.407 g/cm^2^) with a T-score of -4.3 (normal range, >-1.0).

### Treatment and follow-up

The patient continued with life-long levothyroxine treatment, at a dose of 175 μg/day, in addition to medication for hypoferric anemia (50 mg iron-dextrin, three times daily) and osteoporosis (0.25 μg calcitriol, once daily) for six months. A computed tomography scan did not identify any evidence of residual tumor. Monthly treatment with 20 mg octreotide acetate was initiated. Following one month of octreotide acetate treatment, the patient’s GH levels decreased to 4.40 ng/ml and at three months, the GH levels were 5.47 ng/ml. Therefore, octreotide acetate treatment was terminated, however, two months later the GH levels increased again to 16.44 ng/ml.

### Genomic DNA extraction

Peripheral venous blood (2 ml) was obtained from the patient and 10 healthy controls. DNA was isolated from the blood using a blood Genome DNA Extraction kit (Takara Biotechnology Co., Ltd., Dalian, China), dissolved in TE buffer and stored at −20°C. The present study was approved by the Human Ethics Review Committee of The First Hospital of Lanzhou University (Lanzhou, China) and the investigations involving human subjects complied with the principles outlined in the 1983 Declaration of Helsinki.

### DNA amplification and mutation detection

Exons 1–10 of the *MEN1* gene were amplified by polymerase chain reaction (PCR). All the amplified genes and the primers used are indicated in Table II. In addition, a 539-bp fragment, including exons 8 and 9 of the gsα gene, was amplified by PCR using the primer sequences as follows: Forward, 5′-GTGATCAAGCAGGCTGACTATGTG-3′ and reverse, 5′-GCTGCTGGCCACCACGAAGATGAT-3′.

The PCR amplification was performed in a total volume of 50 μl containing 2 μl extracted DNA, 20 pmol of each of the forward and reverse primers, 19 μl 2× Taq PCR Master Mix (Takara Biotechnology Co., Ltd.) and 25 μl deionized water. The PCR cycling conditions were as follows: Initial activation of the DNA polymerase at 95°C for 5 min, followed by 30 cycles at 95°C for 30 min, 52–65°C for 30 min and 72°C for 45 min, and a final extension of 72°C for 5 min. The PCR products were purified and directly sequenced to detect gene mutations, and the sequence results were compared with the normal sequences of the *MEN1* or gsα genes obtained from GenBank.

## Results

A base G was shown in healthy controls at nucleotide 7848 within exon 10 of the *MEN1* gene (Fig. 1A), however, a G→A mutation was identified in the present patient at nucleotide 7848 within exon 10 of the *MEN1* gene (Fig. 1B). The heterozygous missense mutation caused the substitution of alanine (GCA) with threonine (ACA) at amino acid position 541 (A541T) of the MEN1 protein. The forward and reverse sequencing results were consistent. In addition, a base G was shown in healthy controls at nucleotide 7997 within exon 10 of the *MEN1* gene (Fig. 1C), however, the patient demonstrated a G→A mutation at nucleotide 7997 within exon 10 of the *MEN1* gene. The mutation was synonymous, therefore, the proline located at amino acid position 590 of the MEN1 protein was unchanged (P590P; Fig. 1D). No other mutation was observed in exons 8 and 9 of the gsα gene of the patient.

## Discussion

The *MEN1* gene consists of 10 exons, from which exons 2–10 encode a 610-amino acid nuclear protein known as menin. Menin is important in the regulation of DNA transcription and replication, cellular apoptosis, the cell cycle and the maintenance of genome integrity (10). A *MEN1* gene mutation has been observed in patients exhibiting MEN1, an autosomal dominant genetic disease that is characterized by the development of primary tumors that involve two or more endocrine tissues within a single patient, including tumors of the parathyroid gland (95% of cases), pancreatic islets (30–80% of cases) and anterior pituitary gland (15–90% of cases). In addition, >25% of MEN1 patients have been reported to develop thyroid tumors, including adenomas, carcinomas and colloid goiters (11). Furthermore, endocrine-inactive tumors, such as lipomas, angiofibromas and collagenomas are frequently identified in MEN1 patients (12).

In total, >400 varying germline mutations have been identified throughout the *MEN1* gene, which indicates that such mutations are not restricted to a specific functional domain (5). The germline mutations identified include ~50% frameshift insertions and deletions, ~20% nonsense mutations, ~20% missense mutations and ~7% splice-site defects, of which the nonsense mutations, as well as many of the frameshift insertions and deletions and the donor-splice site mutations are loss-of-function truncating mutations involving the menin protein. However, a definitive genotype-phenotype correlation has yet to be established. The proposed mechanism linking *MEN1* mutations with tumor formation involves disruption of the interactions between menin and other proteins, such as activating protein-1 (AP-1), transcription factor Jun D or nuclear factor-κB (NF-κB) to suppress Jun-mediated or NF-κB-mediated transcriptional activation, and between members of the Smad family, Smad3 and the Smad 1/5 complex, ultimately resulting in modified cell cycle regulation and proliferation (13,14).

GH-producing tumors causing acromegaly occur in 3–6% of MEN1 patients (15), and an increased female-to-male ratio in MEN1 patients with pituitary adenoma and acromegaly is observed in familiar and sporadic cases (16). The patient in the present study developed pituitary somatotroph adenomas and papillary thyroid carcinoma without the other tumors commonly associated with MEN1, such as parathyroid, intestinal pancreatic endocrine or adrenal cortical tumors. However, genetic analysis revealed a G→A missense mutation at nucleotide 7848 within exon 10 of the *MEN1* gene, which resulted in the substitution of alanine with threonine at amino acid 541 (A541T) of the menin protein. The present study proposes that the patient’s clinical manifestations may be typical of MEN1 as opposed to pure endocrine tumors; with the presence of subcutaneous fibroma being a specific and unusual clinical manifestation of MEN1. Therefore, a long-term follow-up is required to identify additional endocrine tumors associated with MEN1.

Various studies have demonstrated the prevalence of gsα mutations in GH-secreting pituitary adenomas varies according to geographical location and genetic background of the population (1–3,7), however, the patient described in the present study demonstrated no mutations in exons 8 and 9 of the gsα gene. Previous studies indicated that the prevalence of gsα mutations in GH-secreting pituitary adenomas varies by the geographical location and the genetic background of the population (7,17).

In conclusion, the present study reported the rare case of a patient with coexisting GH-producing pituitary tumors causing acromegaly, papillary thyroid carcinoma and subcutaneous fibroma. Despite pituitary surgery, Gamma-Knife radiosurgery and octreotide acetate treatment, the patient’s GH levels were elevated with no evidence of a residual pituitary tumor upon computed tomography scans. Genetic analysis identified a G→A missense mutation at nucleotide 7848 within exon 10 of the *MEN1* gene, which caused the substitution of alanine by threonine at amino acid 541 (A541T) of menin. Therefore, the pituitary adenomas and thyroid carcinoma exhibited by the present patient may be considered as early manifestations of MEN1 as opposed to pure endocrine tumors. Although there is currently no evidence of other types of tumors associated with MEN1, including parathyroid, intestinal pancreatic endocrine or adrenal cortical tumors, long-term follow-up is necessary.

## Figures and Tables

**Figure 1:** Partial sequencing results of the polymerase chain reaction products of exon 10 in the *MEN1* gene at nucleotide 7848: (A) Normal controls, homozygote GG; and (B) patient, heterozygous GA (G7848A); and at nucleotide 7997: (C) Normal controls, homozygote GG; and (D) patient, heterozygous GA (G7997A). Arrows indicate base locations of the mutations.

**Table I:** Laboratory analysis results.

Parameter	Value	Normal value range
Hemoglobin, g/l	87.00	110–150
Erythrocyte, 10^12^/l	2.79	3.5–5.0
Leukocyte, 10^9^/l	4.44	4.0–10.0
Folic acid, ng/ml	14.80	3.1–17.5
Vitamin B12, pg/ml	403.90	211–946
Serum iron, μmol/l	6.60	9.0–27.0
Unsaturated iron binding capacity, μmol/l	72.40	31–51
Total iron-binding capacity, μmol/l	79.00	54–77
Iron saturation	0.08	0.15–0.55
Ferritin, ng/ml	7.00	13.0–150.0
Serum calcium, mmol/l	2.25	2.10–2.80
Serum phosphorus, mmol/l	1.67	0.97–1.60
Intact parathyroid hormone, pg/ml	24.70	14–72
2,5-hydroxy vitamin D, nmol/l	65.43	47.7–144.0
Osteocalcin, ng/ml	41.60	12.8–55.0
Bone-specific alkaline phosphatase, μg/l	17.50	7.3–22.4

**Table II:** Primers and length of the *MEN1* gene amplification.

Exon	Forward primer (5′→3′)	Reverse primer (5′→3′)	Length, bp	Annealing temperature, °C
2A	TCCCTCCCCCGGCTTGCCTT	ACGTTGGTAGGGATGACGCG	220	60
2B	TGCTGGGCTTCGTGGAGCAT	GAGACACCCCCTTCTCGAGG	220	57
2C	GCCCGCTTCACCGCCCAGAT	GGAGGGTTTTGAAGAAGTGG	230	58
3	TCATTACCTCCCCCTTCCAC	AGGCTGGGGGGAGGGAACAA	254	60
4	AGGGTGGGCCATCATGAGAC	TAGCCCAGTCCTGCCCCATT	207	60
5,6	CATAACTCTCTCCTTCGGCT	TCTGCACCCTCCTTAGATGC	260	60
7	GGATCCTCTGCCTCACCTCC	GCAGGCCCTAGTAGGGGGAT	189	63
8	AGAGACCCCACTGCTCTCACA	GGACACAGGCTGGAGCTCC	187	64
9	AGAGACTGATCTGTGCCCTC	AGACCTCTGTGCAGCTGTCC	227	62
10A	ACGGGCTTGTCAGACTTTTC	ATGCCCTTCATCTTCTCACTC	498	64
10B	GCCAGCACTGGACAAGGGCC	CAGCAGCTCCTTCATGCCCT	205	65
10C	GGGTCCAGTGCTCACTTTCC	CAAGCGGTCCGAAGTCCCCA	218	63
